The article "Analysis of the pattern recognition algorithm of broadband satellite modulation signal under deformable convolutional neural networks" was retracted in 2025. Reasons: compromised peer review; unreliable results or conclusions; concerns about the peer review.

# Analysis of the pattern recognition algorithm of broadband satellite modulation signal under deformable convolutional neural networks

**DOI:** 10.1371/journal.pone.0234068

**Published:** 2020-07-13

**Authors:** Hui Li, Ming Li

**Affiliations:** National Intellectual Property Administration, Beijing, China; University College London, UNITED KINGDOM

## Abstract

This research aims to analyze the effects of different parameter estimation on the recognition performance of satellite modulation signals based on deep learning (DL) under low signal to noise ratio (SNR) or channel non-ideal conditions. In this study, first, the common characteristics of broadband satellite modulation signal and the commonly used signal feature extraction algorithm are introduced. Then, the broadband satellite modulation signal pattern recognition model based on deformable convolutional neural networks (DCNN) is built, and the broadband satellite signal simulation is conducted based on Matlab software. Next, the signal characteristics of binary phase shift keying (BPSK), quadrature phase shift keying (QPSK), 8 phase shift keying (PSK), 16 quadratic amplitude modulation (QAM), 64QAM, and 32 absolute phase shift keying (APSK) are extracted by the constellation map, and the ratio changes of T_1_ and T_2_ with SNR are compared. When SNR is given, it is compared with VGG model, AlexNet model, and ResNe model. The results show that the constellation points of satellite signals with different modulations are evenly distributed. T_1_ of PSK modulation signals increases significantly with the increase of SNR. When SNR is greater than 10, PSK modulation signals can be identified. When T_2_ is set and SNR is greater than 15dB, 16QAM and 32APSK signals can be distinguished. In the model, the Relu activation function, mini-batch gradient descent (MBGD) algorithm, and Softmax classifier have the best recognition accuracy. PSK modulation signals have the best recognition rate when the SNR is 0dB, and the recognition accuracy of different modulation signals at 20dB is over 98%. When the data length reaches 4000, the recognition accuracy of different modulation signals is higher than 97%. Compared with other algorithms, this algorithm has the highest recognition accuracy (99.83%) and shorter training time (3960s). In conclusion, the broadband satellite modulation signal pattern recognition algorithm of DCNN constructed in this study can effectively identify the patterns of different modulation signals.

## 1. Introduction

Nowadays, the development of communication technology shows the trend of rapid growth, and the traditional ground communication technology can’t meet people's daily needs gradually, so more and more experts and scholars focus on the research of satellite communication technology. At present, satellite communication technology has been applied to national defense and people's livelihood, but information interference and other problems have become more and more prominent [1]. Different satellites with the same transmitting signal frequency will interfere with each other, the satellites will also be interfered by the outside world when transmitting signals, and the radiation from some ground facilities will also cause electromagnetic interference to the signals, etc. [2]. When improving the performance of satellite communication system, the recognition of satellite communication modulation mode is the key, but the modulation mode of different signals needs to be determined according to the current channel environment. In the limited space, the density of satellite signals has been greatly increased, so in order to increase the carrying capacity of satellite signals, it is necessary to use different modulation methods for signal modulation. The recognition technology of modulation signals is between receiving and demodulating. After receiving the satellite signals, the method of extracting the modulation signals from the noisy signals can lay a foundation for the subsequent demodulation, parameter estimation, and signal information extraction of the satellite signals [3].

Deep learning can extract the underlying features and integrate them to obtain the high-level features. After adding attribute categories of features, the feature distribution characteristics of the target object can be studied [4]. Moreover, the deep learning model has a strong ability to fit the characteristics of data (Hossain et al., (2019)). In recent years, many studies have shown that machine learning or neural network can be applied to signal feature extraction or signal pattern recognition, but the actual application process will be affected by the change of SNR [5, 6]. The recognition of modulation signals by deep learning algorithm has high robustness, and the recognition types are also very comprehensive. But in the practical application, it will be difficult to realize because of the complexity of the algorithm. Therefore, it is of great significance to construct a modulation signal pattern recognition model with good generalization and large dynamic SNR. However, it is a great challenge to automatically recognize the characteristic parameters, the recognition algorithm, and the modulation method of the classifier in the modulation signal effectively, and to apply it to the recognition of the modulation signal pattern. Therefore, in this study, the DCNN in DL is used to identify the modulation signal pattern of broadband satellite, so as to lay a foundation for the recognition of modulation signal pattern in different SNR environments.

## 2. Literature review

### 2.1. Research status of DCNN

CNN is a deep feedforward artificial neural network model, which has been widely used in the field of image recognition. The DCNN network refers to the application of CNN network for identification research under the condition of variable operation, and it has been widely used in the field of identification. Zhu et al. (2018) applied deformable convolutional neural networks (DCNN) to the recognition and classification of hyperspectral images, and found that this model had higher classification performance than other classification models [7]. Cao et al. (2020) used DCNN model for target recognition and regional regression, and found that the accuracy and recognition speed of the model had significant advantages [8]. Ma et al. (2018) proposed a multi-view convolutional neural network based on DCNN and applied it to image classification to find obvious advantages [9]. Chen et al. (2019) proposed a matrix decomposition model based on DCNN and applied it to text data recommendation. The results showed that the model can effectively improve the accuracy of recommendation [10]. On the whole, DCNN model has a strong advantage in the field of image classification and recognition, but there is no relevant research on the application of DCNN model in satellite modulation signal recognition.

### 2.2. Research status of modulation signal recognition

The identification of early modulation methods is mainly to change the received signal from high frequency to low frequency, demodulate through demodulator, and finally identify the modulation mode through manual methods. Sheng Hong et al. (2019) proposed a signal modulation recognition algorithm based on DL and applied it to the signal recognition of orthogonal frequency-division multiplexing (OFDM) systems. It was found that the proposed method had higher accuracy and consistency than the traditional algorithm for signal extraction [11]. Yu Wang et al. (2019) constructed an automatic modulation recognition algorithm for cognitive radio with CNN, applied it to the recognition of 16 and 64 quadratic amplitude modulation (QAM), and found that the model could be used to classify QAM signals even when the signal intensity was low [12]. Zufan Zhang (2019) et al. proposed an automatic modulation classification method based on the CNN model. After applying it to the classification of spectrum monitoring and cognitive radio, they found that the classification accuracy could reach 92.5% when the SNR was -4db [13]. Sai Huang et al. (2019) proposed a recognition method for automatic modulation classification of signals based on grid constellation matrix and full convolutional network. The results showed that the algorithm had better classification performance, higher robustness, and lower training time [14]. Furui Wang et al. (2019) proposed a vibration tone system method based on nonlinear ultrasonic characteristics, applied it to the monitoring of bolt joints, and found that the model could solve such problems as energy dissipation and low SNR ratio [15]. Yingkun Huang et al. (2019) proposed a feature recognition algorithm for automatic modulation recognition of radar signals, applied it to the recognition of different modulation patterns, and found that the algorithm was almost unaffected by the signal pulse width, and would have high recognition effectiveness and robustness [16]. To solve the problems of modulation classification and symbol decoding, Ertan Kazikli and others (2019) proposed modulation recognition methods based on Bayesian framework and Minimax framework respectively. It was found that compared with conventional technologies, the proposed algorithm could effectively improve the introduced symbol detection performance index [17]. Ade Pitra Hermawan et al. (2020) constructed an automatic modulation classification network based on CNN and applied it to the classification of modulation types of wireless signals, and found that this method improved the classification accuracy and time [18].

To sum up, it can be concluded that the DCNN has better recognition efficiency, and the application of CNN model to the recognition of modulation signal pattern can improve the accuracy of recognition and classification. However, in the existing researches, the recognition of modulation signal pattern is mainly focused on the recognition of radio or radar signals, while there are relatively few researches on the recognition of modulation pattern of satellite signals and the influence of SNR interference on the recognition accuracy. Therefore, in this study, to fill the research gap, the DCNN model is constructed and applied to the recognition of broadband satellite modulation signal patterns, and the effects of different activation functions, descent algorithms, classifiers, and SNR ratios on model recognition rates are compared. It is intended to provide a theoretical basis for improving the recognition accuracy of broadband satellite modulation signal patterns.

## 3. Methodology

### 3.1. Common broadband satellite modulation signals

When PSK is used for signal transmission, it is mainly achieved by changing the phase of the carrier. The signal in BPSK only has two phase values, so the calculation equation of the signal in the time domain is as follows.

$$e_{2PSK}\left(t\right)=\left[\sum_{n}a_{n}g\left(t-nT_{s}\right)\right]\cos\left(\omega_{c}t+\varphi_{n}\right)$$ (1)

Where, *a*_*n*_ is the electrical average value of the bipolar digital signal of the *n*th symbol; *g*(*t*) is the pulse waveform of the base band; *T*_*s*_ is the time width maintained by the symbol (0 or 1); *ω*_*c*_ is the frequency of the carrier angle; *φ*_*n*_ is the absolute phase value of the *n*th symbol.

The expression of QPSK signal is as follows.

$$s_{i}\left(t\right)=A\cos\left(w_{c}t+\theta_{i}\right)$$ (2)

In the equation, t is the sampling interval; *θ*_*i*_ is the phase of the sinusoidal carrier.

The mathematical expression of 8PSK signal is as follows.

$$e\left(t\right)=I\left(t\right)\omega_{c}t-Q\left(t\right)\omega_{c}t=\sqrt{I^{2}\left(t\right)+Q^{2}\left(t\right)}\left(\omega_{c}t+\theta_{n}\right)$$ (3)

In the equation, $\theta_{n}=\frac{{}_{-1}Q\left(t\right)}{I\left(t\right)}$.

QAM is a method applied to signal amplitude and phase keying. The general equation of the signal is as follows.

$$e_{QAM}\left(n\right)=\sum_{i=1}^{N}\sqrt{s_{i}}A\cos\left(\omega_{c}nT+\varphi_{i}+\theta \right)g_{T}\left(nT-iT\right)$$ (4)

Where, $s_{i}=A_{i}^{2}+B_{i}^{2}$. Here, *A*_*i*_ and *B*_*i*_ refer to the quadrature carrier of the same frequency with independent baseband waveforms, and *A*_*i*_,*B*_*i*_,∈{2*m*−1−*M*|*m* = 1,2,⋯,*M*}, $\varphi_{i}=\tan^{-1}\frac{B_{i}}{A_{i}}\mathrm{mod}\left(2\pi \right)$.

The mathematical expression of APSK signal set is as follows.

$$x=r_{k}\exp\left(\frac{2\pi }{n_{k}}i_{k}+\theta_{k}\right)$$ (5)

In the equation, k is the number of concentric circles; r_k_ is the radius of the kth concentric circle; n_k_ represents the number of signal points on the kth concentric circle.

### 3.2. Feature extraction method of broadband satellite modulation signal

The common methods of modulation signal feature extraction include wavelet transform, constellation map, and neural network. Wavelet analysis can realize partial analysis of signals in time domain and frequency domain, and adjust the resolution of signals in time domain and frequency domain adaptively [19]. The calculation equation of the general continuous wavelet transform is as follows.

$$WT_{s}\left(b,a\right)=\frac{1}{\sqrt{a}}\int_{-\infty }^{+\infty }s\left(t\right)g^{*}\left(\frac{t-b}{a}\right)dt=\left[s\left(t\right),g_{\left(b,a\right)}\left(t\right)\right]$$ (6)

Where, a and b are scale and displacement factors respectively, and *g*(*t*) is the basis function of the wavelet, S(t) is the orthogonal component.

Neural network can extract the classification features of signals through continuous iterative learning. Assuming that the mean value of signals that can be received is 0 and the variance is 1, then the calculation equation of feature vector $f_{i}^{'}$ is as follows.

$$f_{i}^{'}=\frac{f_{i}-\frac{1}{M}\sum_{j=1}^{M}f_{i}^{\left(j\right)}}{\sqrt{\frac{1}{M}\sum_{j=1}^{M}{\left|f_{i}^{\left(j\right)}-\frac{1}{M}\sum_{j=1}^{M}f_{i}^{\left(j\right)}\right|}^{2}}}$$ (7)

In the above equation, M is the training sample set. After the normalization of the feature vectors, they are input into the neural network, and the final prediction results are output through the calculation of the feedforward network.

$$y_{k}=\frac{\exp\left(a_{k}\right)}{\sum_{j}\exp\left(a_{j}\right)}$$ (8)

Where, *a*_*j*_ is the activation of the *j*th node in the output network.

In this study, the constellation map is mainly used to extract the features in the satellite signal. Assuming that the data quantity of the satellite signal is N and the number of grid squares in the constellation map is k, then the probability of constellation points falling into a grid is as follows.

$$p_{i}=\frac{n_{i}}{N},\;i=1,2,\cdots ,k$$ (9)

In the above equation, *n*_*i*_ is the number of constellation points in each grid.

Constellation map is one of the methods for feature extraction and recognition in modulation signals, which is mainly a vector map obtained in I and Q two-dimensional coordinates by projecting specific basis vectors to the endpoints. When frequency offset and noise exist in the constellation map, the distribution state of constellation points in the diagram is also inconsistent, so the characteristic parameter T_1_ needs to be used to distinguish the amplitude-phase modulation signals in the constellation map, and T_1_ = D(P). Since the constellation maps of QAM and APSK signals are images of multiple rings and the number of rings of different signals is different, the identification of the two signals needs to be distinguished by the characteristic parameter T_2_, and T_2_ = E(丨x_i_丨).

### 3.3. Broadband satellite modulation signal model and preprocessing

The broadband satellite modulation signals to be identified include 6 kinds of signals, that is, BPSK, QPSK, 8PSK, 16QAM, 64QAM, and 32APSK. The baseband signal analysis equation of the signal modulation mode set is as follows.

$$r\left(kT_{s}\right)=e^{j\left(2\pi \Delta fkT_{s}+\theta \right)}\sum_{n}a_{n}g\left(kT_{s}-nT-\varepsilon T\right)+v\left(kT_{s}\right)$$ (10)

In the above equation, Δ*f* is the amplitude of frequency swing of frequency modulation wave of the remaining carrier; *θ* is the initial phase of the carrier; T is the period of the modulation signal; *T*_*s*_ is the sampling period of the modulation signal; *g*(*kT*_*s*_) is the function of the equivalent filter; *ε* is the timing error of the modulation signal; *v*(*kT*_*s*_) is the compound white gaussian noise whose mean value is 0 and the variance value is σ_n_^2^; and *a*_*n*_ is the signal sequence after homogeneous processing.

The calculation equations of MPSK, MQAM, and MAPSK in the mode set are as follows.

$$\left\{ \begin{array}{l} a_{n}=e^{j\left(2i+1\right)\pi /M},\;i=0,1,\cdots ,M-1,\;M=2,4,8\\ a_{n}=A_{M}\left(I_{n}+jQ_{n}\right),\;I_{n},Q_{n}=2i-\frac{M}{4}+1,\;M=16,64\\ a_{n}=r_{k}\exp\left[j\left(\frac{2\pi }{n_{k}}i_{k}+\theta_{k}\right)\right] \end{array}\right.$$ (11)

32 APSK signal can be calculated in the form of 4+12+16APSK, and *r*_3_:*r*_2_:*r*_1_ = 5.27:2.84:1. Then, in this study, symbol rate estimation of broadband satellite signals is carried out, and the main steps are as follows. First, the square processing of the broadband satellite signal modulus is performed, and Fast Fourier transform (FFT) is performed to calculate the modulus square spectrum in the signal. Second, the spectral line of sign rate is searched in the range of sampling frequency.

### 3.4. Construction of the model for pattern recognition of broadband satellite modulation signal based on DCNN

With the rapid development of satellite communication technology, this technology has been widely applied to various fields of the society, and the signals received on the receiver can only be applied to daily life after decoding, modulation, recognition, and channel decoding [20]. Therefore, modulation pattern recognition of satellite signals has become the focus of research. The structure of common broadband satellite communication system is shown in Fig 1, which mainly includes satellite, monitoring and management station, tracking telemetry and command station, communication gateway station, ground communication network. and terminal, etc.

**Fig 1:** Broadband satellite communication system.

In this study, DCNN is used to construct a pattern recognition algorithm for broadband satellite modulation signals. The main recognition process is as follows. First, satellite signals to be trained are input. Second, DCNN is applied to construct network model. Third, the predicted satellite signal is input into the network model and the modulation mode is output. In this study, the basic structure of DCNN is shown in Fig 2.

**Fig 2:** Basic structure of DCNN.

It can be observed from Fig 2 that satellite signal images are input into the network, and the image size of the input layer is 64*64. The variable convolution layer contains 4 convolutional networks and 4 filters for image training. The size of convolution kernel is 3*3. After the output of 4 characteristic graphs of 60*60, they are input to the pooling layer. The size of convolution kernel in pooling layer is 2*2, and the size of output characteristic graph is 30*30. Finally, through the fully connected layer, the classifier is included in the output. In this study, variable learning rate is also introduced into DCNN, and Adam adaptive learning rate is mainly used to estimate sparse data.

In DCNN, the activation function has a greater impact on the accuracy of signal recognition, and the commonly used activation functions include Sigmoid, Tanh, Relu, Leaky Relu, Exponential linear units (ELU), and MaxOut, etc. [21, 22]. Gradient descent in the network can adjust network back propagation parameters, while the commonly used gradient descent algorithms are stochastic gradient descent (SGD), batch gradient descent (BGD) and MBGD [23]. Classifiers for image classification during output include Softmax, Logistic, Boosting, Adaboost, SVM [24]. In this study, Matlab software is used for the simulation of broadband satellite signals, and the characteristic parameters T_1_ and T_2_ of different signals are compared with the changes of SNR. The parameters in the DCNN are adjusted to set the carrier frequency as 640Hz, the symbol speed as 40Hz, the signal sampling frequency as 5200Hz, the number of sampling points as 2000, and the SNR as -12, -8, -4, 0, 4, 8, 12, and 16dB. Different signals are adopted to construct the training set containing 1500 samples and the verification set containing 100 samples. The data length of the signal is set as 2000 symbol, the SNR is between 0 and 20dB, the step-size parameter is 1dB, and the average recognition rate of different signals is calculated. The SNR of different signals is set as 20dB, and the data length of signals is set as 1000–5000 to calculate the average recognition rate of different signals. And the recognition performance of the proposed algorithm is compared with that of other algorithms.

## 4. Results

### 4.1. Constellation characteristics of different broadband satellite modulation signals

It can be observed from Fig 3 that the number of constellation points of each ring of BPSK, QPSK, 8PSK, 16QAM, 64QAM, and 32APSK is {2}, {4}, {8}, {4, 8, 4}, {4, 8, 4, 8, 8, 12, 8, 84}, and {4, 12, 16}. In the case of SNR of 20dB, constellation maps of different modulation signals without frequency deviation have a common characteristic, that is, the different points are distributed in concentric circles with the same radius, the constellation points of different signals are evenly distributed, and the boundaries between the constellation points are clear.

**Fig 3:** Constellation map of different modulation signals.

### 4.2. Variation of characteristic parameters and SNR of different broadband satellite modulation signals

In the presence of noise or frequency offset, the constellation map of different modulation signals will change differently. Therefore, in this study, characteristic parameters T_1_ and T_2_ of modulation signals are introduced to distinguish different signals, and the corresponding changes of characteristic parameters are compared when SNR changes, as shown in Fig 4. It can be observed from Fig 4A that the characteristic parameter T_1_ of BPSK, QPSK, and 8PSK modulation signals increases significantly with the increase of SNR, and PSK modulation signals can be identified when the SNR is greater than 10. And the characteristic parameter T1 of the 16QAM modulation signal will decrease first and then increase as the SNR increases. The characteristic parameters T_1_ of 64QAM and 32APSK modulation signals will gradually decrease as the SNR increases. It can be observed from Fig 4B that the characteristic parameter T_2_ of different modulation signals increases gradually with the increase of SNR, while BPSK, QPSK, 8PSK, 16QAM, 64QAM, and 32APSK signals can be distinguished when SNR is greater than 15dB.

**Fig 4:** Variation curves of characteristic parameters of different modulation signals with SNR.

### 4.3. Performance test of broadband satellite modulation signal recognition model based on DCNN

The influence of different activation functions, gradient descent algorithm, and classifier on the accuracy of signal pattern recognition model based on DCNN is compared. As can be observed from Fig 5A, Sigmoid activation function and Tanh activation function have low recognition accuracy, while Leaky Relu, ELU, and MaxOut activation functions show little difference in recognition accuracy between the signal pattern recognition model based on DCNN constructed in this study. In the model, Relu activation function and Softmax classifier are used to compare the effects of different gradient descent algorithms on the recognition accuracy. It can be observed from Fig 5B that the constructed model has with high recognition accuracy after BGD and MBGD algorithms are applied. And Relu activation function and MBGD descending algorithm are used in the model to compare the influence of different classifiers on the recognition accuracy. It can be observed from Fig 5C that the model recognition accuracy of Softmax classifier is the best.

**Fig 5:** Influence of different parameter settings on the accuracy of model recognition.

Relu activation function, MBGD descent algorithm, and Softmax classifier are used to set the parameters of the constructed model in this study, and the effects of different SNR on the recognition accuracy of different modulation signals are compared. As can be observed from Fig 6, with the increase of SNR, the recognition accuracy of different modulation signals also gradually increases, and when the SNR is 20dB, the recognition accuracy of all modulation signals reaches the maximum value. When SNR is 0dB, the recognition accuracy of BPSK, QPSK, 8PSK, 16QAM, 64QAM, and 32APSK is 96.88%, 93.49%, 90.64%, 85.35%, 57.26%, and 30.12%, respectively. When the SNR is 20dB, the recognition accuracy of BPSK, QPSK, 8PSK, 16QAM, 64QAM, and 32APSK is 100%, 99.81%, 99.54%, 98.97%, 98.85%, and 98.13%, respectively.

**Fig 6:** Variation of recognition accuracy of modulation signals at different SNR.

The SNR is set as 20dB to test the influence of different data lengths on the identification accuracy of the model constructed in this study when the data length is 1000–5000. It can be observed from Fig 7 that when the data length is 1000–2500, the identification accuracy of BSPK, QSPK, and 8SPK modulation signals is higher than that of 16QAM, 64QAM, and 32APSK. And when the data length is 1000, the recognition accuracy of BSPK, QSPK, and 8SPK modulation signals is 80.21%, 80.88%, and 82.89%, respectively. When the data length increases to 3000, the recognition accuracy of 32ASPK modulation signal reaches 99.51%. When the data length reaches 4000, the recognition accuracy of BPSK, QPSK, 8PSK, 16QAM, 64QAM, and 32APSK is 100.00%, 99.97%, 99.91%, 97.13%, 99.10%, and 99.75%, respectively.

**Fig 7:** Variation of recognition accuracy of modulation signals with different data lengths.

The performance of modulation signal recognition was compared with that of VGG model, AlexNet model and ResNet model. As can be seen from Table 1, the recognition accuracy of the model constructed in this study is the highest (99.83%), and the training time is relatively short (3960s).

**Table 1:** Comparison of recognition performance of different models.

Performance	VGG	AlexNet	ResNet	Our Model
Accuracy (%)	99.31	99.42	99.80	99.83
Training time (s)	7200	3600	17280	3960

## 5. Discussion

High-speed satellite data transmission requires the use of high modulation dimension and the number of multiple constellation points. Based on constellation map, the features in the signal can be effectively extracted. Therefore, in this study, first, the constellation map is used to extract the features of broadband satellite signals. The results show that the different points in the constellation map of different modulation signals are distributed in concentric circles with the same radius. Then the constellation map is used as the input sample for the pattern recognition of DCNN satellite modulation signals constructed in this study, and the changes of different characteristic parameters in the constellation map with the increase of SNR are compared. The results show that PSK modulation signal patterns can be effectively identified when the SNR is greater than 10dB, which is basically consistent with the results of Mohamed Al-Nahhal et al. (2019) [25]. Next, in this study, the effects of different activation functions on the recognition accuracy of the constructed model are compared. It is found that the DCNN model based on Leaky Relu, ELU, and MaxOut activation functions have higher recognition accuracy, the calculation of Leaky Relu activation function is relatively simple, and its convergence rate is faster than that of Sigmoid and Tanh activation function [26]. However, the most classical activation function is Relu, and the recognition accuracy of the model based on Relu activation function is higher than that of Sigmoid activation function [27]. Therefore, in this study, Relu activation function is adopted for subsequent experiments. The influence of different gradient descent algorithms on the recognition accuracy of the model constructed in this study is compared, and it is found that the model recognition accuracy based on BGD and MBGD descent algorithm is relatively high, which is basically consistent with the results of Wenbin Jiang et al. (2020) [28]. However, the calculation speed of BGD is slow and new data can’t be input to update the model in real time. SGD algorithm is updated too frequently, which will cause shock of cost function. While MBGD can reduce the variance when parameters are updated, and the convergence is stable. It can use the height optimization matrix in DL for gradient calculation [29, 30]. Therefore, MBGD algorithm is selected for subsequent research. The results of the influence of different data lengths on the recognition accuracy of the model show that in the recognition of modulation signals, only when the length of data exceeds 4000, can a good recognition accuracy be achieved. Too small data lengths are not conducive to the recognition of 16QAM, 64QAM, and 32APSK modulation signals. Compared with VGG [31], AlexNet [32], and ResNet [33] models, the identification accuracy of the model constructed in this study is higher.

## 6. Conclusions

The purpose of this research is to improve the accuracy rate of pattern recognition of satellite modulation signals under low SNR or unsatisfactory channel conditions. In this study, it is found that when feature extraction of satellite signal is carried out with constellation map, PSK modulation signals can be effectively recognized when SNR is 10dB. When constructing the DCNN model to identify the broadband satellite modulation signal pattern, the application of Relu activation function, MBGD descent function, and Softmax classifier can achieve high recognition accuracy. When the SNR is greater than 15dB and the data length is greater than 3500, it can effectively identify different modulation signal patterns, and the overall recognition accuracy of the model constructed in this study can reach 99.83%. However, in this study, only the influence of different parameter settings on the accuracy of pattern recognition of modulation signals is studied. Since satellite transmission signals contain a large amount of data, further research on signal image compression and storage is needed. In a word, the recognition algorithm of broadband satellite modulation signal pattern based on DCNN constructed in this study can effectively improve the satellite signal of different debugging modes and lay a foundation for solving the interference of satellite signal transmission.

## Supporting information

S1 Data (XLSX)

S1 Code (DOC)
